The article "Impacts of Low-Dose Total Glycosides of Tripterygium wilfordii plus Methotrexate on Immunological Function and Inflammation Level in Patients with Rheumatoid Arthritis" was retracted in 2023. Reasons: unreliable results or conclusions; concerns about the data; concerns about the peer review; concerns about the citations.

# Impacts of Low-Dose Total Glycosides of Tripterygium wilfordii plus Methotrexate on Immunological Function and Inflammation Level in Patients with Rheumatoid Arthritis

**DOI:** 10.1155/2022/7523673

**Published:** 2022-08-01

**Authors:** Yong Han, Jingri Jin, Fushun Wu, Zhiwei Wang

**Affiliations:** ^1^Department of Immunology, Yanbian University Hospital, Yanji, 133000 Jilin, China; ^2^Department of Osteology, Yanbian University Hospital, Yanji, 133000 Jilin, China

## Abstract

**Purpose:**

This research mainly clarifies the impacts of low-dose- (LD-) total glycosides of Tripterygium wilfordii (GTW) plus methotrexate (MTX) on immunological function and inflammation level in patients with rheumatoid arthritis (RA).

**Methods:**

We enrolled 106 RA patients treated in Yanbian University Hospital between July 2019 and July 2021, including 56 cases (research group) intervened by LD-total GTW plus MTX and 50 cases (control group) treated with MTX, in addition to conventional treatment given to both groups. The improvement in immunological function (immunoglobulin (Ig) A, IgG, and IgM), inflammatory cytokines (ICs; C-reaction protein (CRP), tumor necrosis factor-*α* (TNF-*α*), and interleukin-6 (IL-6)), incidence of adverse reactions (ARs), joint function, and patient satisfaction were observed and compared.

**Results:**

Statistical better improvements of immunological function, ICs, and joint function were observed in the research group compared with the control group. Besides, patient satisfaction was higher and the incidence of ARs was lower in the research group.

**Conclusions:**

LD-total GTW plus MTX is highly effective and safe in enhancing the immunity, lowering the inflammation level, and improving the joint function of RA patients.

## 1. Introduction

Rheumatoid arthritis (RA), one of the most commonly seen chronic inflammatory diseases, is a chronic autoimmune condition affecting joints. It is characterized by progressive and symmetrical inflammation of the affected joints, leading to cartilage destruction, bone erosion, and ultimately disability [1]. In the later stages of the disease, many joints are involved with extra-articular symptoms in most cases [2]. The incidence of RA varies by gender, age, and patient group [3]. The prevalence of this connective tissue disease, which is associated with reduced quality of life, poor functional status, and increased mortality, has increased over the past two decades, further increasing the disease burden [4]. The condition of RA is prone to fluctuate with the aggravation of episodes. Without optimal treatment, the patient's symptoms can progressively worsen until the joints are irreversibly damaged and physical and mental functions are affected [5]. In addition, the complications and comorbidities of RA can reduce life expectancy by several years [6, 7]. For these reasons, the treatment of RA needs a careful selection. In this study, we take drugs such as total glycosides of Tripterygium wilfordii (GTW) and methotrexate (MTX) as examples to study the drug treatment of RA, aiming to provide new reference for the treatment of RA and the improvement of patients' condition.

The article "Impacts of Low-Dose Total Glycosides of Tripterygium wilfordii plus Methotrexate on Immunological Function and Inflammation Level in Patients with Rheumatoid Arthritis" was retracted in 2023. Reasons: unreliable results or conclusions; concerns about the data; concerns about the peer review; concerns about the citations.

Tripterygium glycosides (TG) are a kind of natural active ingredient extracted from Tripterygium wilfordii, a southern Chinese vine that has long been used in traditional Chinese medicine [8]. Due to diverse pharmacological effects such as detoxification, blood-activating, inflammation prevention, and antiprocreation, the drug has been widely used to treat various types of inflammation [9]. It works by inhibiting dihydroorotate dehydrogenase, even in the treatment of active moderate-to-severe RA [10]. Another long widely used drug for severe RA, MTX, inhibits inflammation by suppressing dihydrofolate reductase. MTX treatment, however, often comes with side effects [11]. Therefore, MTX needs to be combined with other drugs during treatment. However, for RA, there are few related studies on the combination treatment of the above two drugs. The purpose of this study is to study the impact of low-dose- (LD-) total GTW combined with MTX on RA patients through immunity- and inflammation-related indicators.

## 2. Methods

### 2.1. General Information

The study population comprised 106 cases of RA treated in Yanbian University Hospital from July 2019 to July 2021. According to different treatment methods, they were assigned to either the control group or the research group. The research group, with 56 cases, was treated with LD-total GTW plus MTX and conventional treatment, while the control group (50 cases) received MTX and routine treatment. The two cohorts showed no significant differences in general data (*P* > 0.05), with comparability. Inclusion criteria are as follows: all patients were diagnosed as RA in our hospital and were mentally normal that could accurately express their discomfort, with no history of drug allergy related to this study. Exclusion criteria are as follows: serious heart, liver, kidney, and other organ diseases; pregnant or lactating woman; use of immunosuppressants within 30 days before enrollment; and missing or incomplete clinical records.

The family members of patients gave their consent for patients' participation in this study and signed the relevant agreement. This study has obtained approval from the Medical Ethics Committee of Yanbian University Hospital.

The article "Impacts of Low-Dose Total Glycosides of Tripterygium wilfordii plus Methotrexate on Immunological Function and Inflammation Level in Patients with Rheumatoid Arthritis" was retracted in 2023. Reasons: unreliable results or conclusions; concerns about the data; concerns about the peer review; concerns about the citations.

### 2.2. Treatment Methods

Both groups received routine treatment. Oral indomethacin (Guangdong Huanan Pharmaceutical Group, SFDA Approval No. H44020701) was administered 0.1 g once, 3 times/d. Additionally, a reasonable diet was adopted, and high-fat and high-cholesterol foods were avoided as much as possible. On this basis, the control group was given 15 mg MTX (SFDA Approval No. H31020644, specification: 2.5 mg × 100 tablets) produced by Shanghai Pharmaceuticals Sine, per os, once a week. The research group was given oral LD-total GTW and MTX. 10 mg total GTW (Jiangsu Meitong Pharmaceutical Co., Ltd., SFDA Approval No. Z32021007) was administrated 3 times per day and 7. 5 mg MTX was given once a week. Both groups were treated for 3 months, and the dosage of indomethacin was halved after 1 month of treatment and stopped after 2 months of treatment.

### 2.3. Measurement Indicators

Before the detection of immunological function and inflammatory cytokines (ICs) in patients, we collected 5 mL of fasting cubital venous blood from patients before and after treatment and extracted serum by 10 min of centrifugation at 1500 × *g* and 4°C.

#### 2.3.1. Immunological Function

Serum immunoglobulins of both cohorts of patients were quantified before and after treatment. Immunoglobulin (Ig) A, IgG, and IgM contents were measured using a spectrophotometer (Shanghai Huicheng Biotech, C001-96T-1).

#### 2.3.2. ICs

Serum ICs in both cohorts were measured before and three days after treatment. C-reaction protein (CRP), tumor necrosis factor-*α* (TNF-*α*), and interleukin-6 (IL-6) concentrations were detected by enzyme-linked immunosorbent assay (ELISA). The assay was carried out strictly following the instructions of the corresponding human ELISA kit (Wuhan Fine Biotech, EH2643, AQ-H0302-B, AQ-H0201).

#### 2.3.3. Incidence of Adverse Reactions (ARs)

The incidence of ARs in the two groups was detected and compared, and the related indicators were nausea, belching, abdominal pain, and mucosal ulcer.

#### 2.3.4. Evaluation of Joint Function

Patients' joint function after treatment was compared. The joint function was evaluated according to the “Joint Dysfunction Grading Standard” [12]: (1) Grade I: patients can carry out daily life and work. (2) Grade II: patients can carry out general daily life and some professional work, but with confined activity. (3) Grade III: patients can carry out general daily life, but cannot participate in certain work or projects, with activity limitations. (4) Grade IV: patients cannot take care of themselves in daily life, with limited working ability.

#### 2.3.5. Patient Satisfaction

We also compared patients' satisfaction with the nursing, using the nursing satisfaction questionnaire with the test contents and evaluation criteria all designed by our hospital. On a 100-point scale, 100-85, 60-84, and below 60 indicated satisfied, 60-84 basically satisfied, and dissatisfied, respectively. Satisfaction = (satisfied cases + basically satisfied cases)/total cases∗100%.

The article "Impacts of Low-Dose Total Glycosides of Tripterygium wilfordii plus Methotrexate on Immunological Function and Inflammation Level in Patients with Rheumatoid Arthritis" was retracted in 2023. Reasons: unreliable results or conclusions; concerns about the data; concerns about the peer review; concerns about the citations.

### 2.4. Statistical Methods

SPSS22.0 (Asia Analytics formerly SPSS China) was used for the statistical processing of comprehensive data. Enumeration data were tested by *χ*^2^, while quantitative data denoted by (*X* ± *S*) were verified by the *t*-test, with *P* < 0.05 as the significance threshold.

## 3. Results

### 3.1. General Information

The research group and the control group were not statistically different in a series of general data such as gender, age, body mass index (BMI) (*P* > 0.05). See Table 1 for details.

### 3.2. Immunological Function

The immunoglobulin levels differed insignificantly between research group and the control group prior to treatment (*P* > 0.05). The posttreatment IgG, IgA, and IgM levels decreased compared with their pretreatment levels, and the improvement of the above indexes was more obvious in the research group (*P* < 0.05; Figure 1).

### 3.3. ICs

Similarly, ICs were not notably different between groups prior to treatment (*P* > 0.05). And statistical decreases were observed in CRP, TNF-*α*, and IL-6 in both cohorts of patients after treatment, with more significant improvement of the above indexes in the research group compared to the control group (*P* < 0.05; Figure 2).

### 3.4. Incidence of ARs

After investigating ARs in the two groups, it was found that the incidence was significantly lower in the research group compared with the control group (*P* < 0.05). Please see Table 2 for details.

### 3.5. Joint Function Evaluation

As shown in Table 3, the proportion of grade I joint dysfunction in the research group increased significantly after treatment compared with the control group (*P* < 0.05), but there was no significant difference between groups in the proportions of grade II and grade III joint dysfunction (*P* > 0.05).

### 3.6. Patient Satisfaction

The investigation of patient satisfaction revealed a higher satisfaction degree in the research group as compared to the control group (*P* < 0.05; Table 4).

## 4. Discussion

As a disease of unknown origin, RA causes inflammatory changes in synovial tissues, cartilage, and hard bones of joints and, less commonly, in the extra-articular sites. Patients with RA mainly present with joint pain, swelling, and subsequent cartilage and bone destruction, as well as systemic manifestations caused by arachidonic acid metabolites and various ICs [13]. There is currently no cure for such a systemic inflammatory disease, and because of its heterogeneity, variability, and multilevel nature, there is no a unified description of its pathogenesis, so the treatment of it is still a difficulty [14]. In this section, we will discuss the impacts of the two-drug combination therapy on the immunological function and inflammation level of RA based on the results obtained.

The article "Impacts of Low-Dose Total Glycosides of Tripterygium wilfordii plus Methotrexate on Immunological Function and Inflammation Level in Patients with Rheumatoid Arthritis" was retracted in 2023. Reasons: unreliable results or conclusions; concerns about the data; concerns about the peer review; concerns about the citations.

According to the results, the research group that used the combination of the two drugs had significantly better immunological function recovery than the control group. In the study of Dong et al. [15], the application of GTW to patients with RA could significantly reduce IgA and IgG levels in patients, similar to our findings. Liu et al. [16] also pointed out that GTW and MTX had significant inhibitory effects on the levels of IgG, IgA, and IgM in RA patients with anemia, which was consistent with our results. A combination therapy of MTX with other drugs can significantly improve patients' immunological function. This is because when combined with other drugs, it inhibits tyrosine kinases that affect immunological function while reducing the production of pyrimidine and dihydroorotate dehydrogenase to inhibit DNA synthesis, enabling it to exert a pharmacodynamic mechanism on lymphocyte activation and immune response, thus enhancing the immunity of patients [17–19]. On the other hand, MTX, when used alone, brings many side effects and has a poor effect on lymphocyte proliferation of the immune system. Therefore, it is necessary to combine with other drugs to inhibit lymphocyte proliferation and finally improve the abnormal immune response of RA patients [20–22]. As an extract of Chinese herbal medicine, total GTW is effective in the treatment of various systemic diseases [23]. Tripterygium glycosides belong to a nonsteroidal immunosuppressant, which can effectively inhibit cellular immunity and humoral immunity [8, 24]. Currently, the drug is extensively used to treat autoimmune diseases, including RA, primary glomerulonephritis, and immune-related nephritis [25, 26]. According to the characteristics of the two drugs, the combination of total GTW can effectively make up for the deficiency of MTX and adjust patients' immunity.

In terms of inflammation, more significantly reduced levels of ICs were determined in the research group after treatment. In the treatment of various types of arthritis, the antifolic acid mechanism of MTX has historically been related to the treatment of neoplastic (lymphoblastic) diseases. The immunosuppression brought by LD-MTX therapy can even play an anticancer role, which mainly depends on the inhibition of the enzyme 5-aminoimidazole-4-carboxamide ribonucleoside (AICAR) transformylase (ATIC), resulting in a higher level of AICAR inhibition of adenosine monophosphate deaminase and adenosine deaminase. This leads to higher extracellular levels of adenine, which is further converted into adenosine, thus playing an anti-inflammatory role through adenosine receptors. It also reduces downstream inflammatory signaling via the nuclear factor kappa B (NF*κ*B) [27]. However, the antifolate effects of MTX also contribute to most of its side effects and result in it having little effect on inhibiting other anti-inflammatory pathways [28], which may explain the limited decrease of ICs in the control group using MTX alone. As mentioned above, Tripterygium wilfordii has anti-inflammatory action, which can be enhanced if MTX is combined. Combining the conclusions of previous literature with our findings, we can conclude that the combination of the two drugs can effectively improve patient's immunological function and relieve inflammation, which can facilitate patients' rehabilitation and improved limb recovery. And because of the combination of the two, the side effects of MTX can even be effectively reduced, contributing to higher patient safety, fewer ARs, and higher patient satisfaction. In the report of Wang et al. [29], GTW plus MTX in patients with RA significantly inhibited the level of CRP without increasing the complication rate, which is consistent with our findings. Wang et al. [30] also pointed out that compared with MTX alone, GTW combined with MTX intervention can significantly improve the clinical manifestations of joint swelling and tenderness in RA patients, indicating higher efficacy of the combined treatment in improving patients' joint function, which can support our results. Chen et al. [31] also reported a higher compliance degree in RA patients treated with GTW and MTX combination therapy compared with those receiving MTX monotherapy, which reflected that the satisfaction rate of RA patients with combined therapy may be relatively higher.

The article "Impacts of Low-Dose Total Glycosides of Tripterygium wilfordii plus Methotrexate on Immunological Function and Inflammation Level in Patients with Rheumatoid Arthritis" was retracted in 2023. Reasons: unreliable results or conclusions; concerns about the data; concerns about the peer review; concerns about the citations.

The innovation of this study lies in the comparative evaluation of the clinical effects of LD-total GTW combined with MTX combined with MTX and MTX monotherapy in the treatment of RA from the perspectives of immunological function, ICs, incidence of ARs, joint function, and patient satisfaction. This study confirmed the efficacy and safety of the combination therapy for patients with RA, providing a new basis for the treatment of such patients. However, there are many shortcomings in this study. We failed to effectively observe patients' treatment compliance during the treatment process nor have we investigated the psychological anxiety and depression of them. In future research, we will continue to address the above deficiencies, and constantly improve the treatment methods to make patients satisfied.

Conclusively, this research believes that LD-total GTW combined with MTX can significantly improve RA patients' immunity, reduce inflammation, and improve their joint function with higher safety.

## Figures and Tables

**Figure 1:** Immunoglobulins of the two groups of patients: (a) IgG levels in the two groups, (b) IgA levels in the two groups, and (c) IgM levels in the two groups. ∗ means *P* < 0.05 compared with before treatment, and # means *P* < 0.05 compared with the control group.

**Figure 2:** Inflammatory cytokines of the two groups of patients: (a) CRP levels in the two groups, (b) IL-6 levels in the two groups, and (c) TNF-*α* levels in the two groups. ∗ means *P* < 0.05 compared with before treatment, and # means *P* < 0.05 compared with the control group.

**Table 1:** General data.

Classification	Research group (*n* = 56)	Control group (*n* = 50)	*t*/*χ*^2^	*P*
Sex			0.03	0.872
Male	30	26		
Female	26	24		
Age (years old)	61.77 ± 7.36	60.84 ± 7.15	0.66	0.512
BMI (kg/m^2^)	26.06 ± 2.87	25.26 ± 2.97	1.41	0.162
Work location			0.40	0.528
Urban areas	38	31		
Rural areas	18	19		
Smoking			0.11	0.743
Yes	41	38		
No	15	12		
Drinking			0.07	0.792
Yes	35	30		
No	21	20		

**Table 2:** Incidence of adverse events.

Classification	Research group (*n* = 56)	Control group (*n* = 50)	*χ* ^2^	*P*
Nausea	2 (3.57)	3 (6.00)		
Eructation	0 (0.00)	1 (2.00)		
Abdominal pain	2 (3.57)	1 (2.00)		
Mucosal ulcer	0 (0.00)	6 (12.00)		
Incidence of adverse reactions (%)	4 (7.14)	11 (22.00)	5.86	0.012

**Table 3:** General data.

Classification	Research group (*n* = 56)	Control group (*n* = 50)	*χ* ^2^	*P*
Grade I	33 (58.93)	19 (38.00)	4.63	0.031
Grade II	18 (32.14)	21 (42.00)	1.10	0.294
Grade III	5 (8.93)	10 (20.00)	2.67	0.103

**Table 4:** Satisfaction of the two groups of patients.

Classification	Research group (*n* = 56)	Control group (*n* = 50)	*χ* ^2^	*P*
Satisfied	36 (64.29)	22 (44.00)	—	—
Basically satisfied	18 (32.14)	18 (36.00)	—	—
Dissatisfied	2 (3.57)	10 (20.00)	—	—
Satisfaction (%)	54 (96.43)	40 (80.00)	7.45	0.006

## Data Availability

The labeled datasets used to support the findings of this study are available from the corresponding author upon request.
